The article "Effects of hsa-miR-28-5p on Adriamycin Sensitivity in Diffuse Large B-Cell Lymphoma" was published in 2022. Journal: Evid Based Complement Alternat Med.

# Effects of hsa-miR-28-5p on Adriamycin Sensitivity in Diffuse Large B-Cell Lymphoma

**DOI:** 10.1155/2022/4290994

**Published:** 2022-07-13

**Authors:** Shufang Yan, Qinyu Shang, Haipeng Zhu, Ken Chen, Xinxia Li, Hongliang Gao, Bo Liu, Mei Feng, Lixia Gao

**Affiliations:** ^1^Department of Critical Care Medicine, Karamay Central Hospital, Karamay City 834000, The Xinjiang Uygur Autonomous Region of China, China; ^2^Department of Pathology, The Tumor Hospital Affiliated to Xinjiang Medical University, No. 789 Suzhou Dongjie, Urumqi 830011, The Xinjiang Uygur Autonomous Region of China, China; ^3^Xinjiang Medical University, No. 567 North Shangde Road, Urumqi 830011, The Xinjiang Uygur Autonomous Region of China, China; ^4^Department of Hematology Oncology of Karamay Central Hospital, Number 67, Junggar Road, Karamay Region, Karamay 834000, The Xinjiang Uygur Autonomous Region of China, China; ^5^Department of Pathology, The First Affiliated Hospital of Xinjiang Medical University, No. 137 Liyushan Southern Road, Urumqi 830054, The Xinjiang Uygur Autonomous Region of China, China; ^6^Department of Emergency of Karamay Central Hospital, Number 67, Junggar Road, Karamay Region, Karamay 834000, The Xinjiang Uygur Autonomous Region of China, China

## Abstract

**Background:**

Adriamycin (doxorubicin) is an important traditional drug that exhibits cytotoxicity in Diffuse Large B-cell Lymphoma (DLBCL). Doxorubicin affects the DLBCL cells at all stages of their cell cycle. Combined with our previous results, this study discovered that the overexpression of hsa-miR-28-5p inhibited the proliferation, promoted apoptosis, and triggered cell cycle arrest at the S-phase in DLBCL cells. However, the effect of (Homo sapiens, hsa)-microRNA (miR)-28-5p on doxorubicin sensitivity in DLBCL has not been investigated. This study aims to reveal the effects of hsa-miR-28-5p on doxorubicin sensitivity at the level of DLBCL cells.

**Methods:**

To determine the optimal concentration of doxorubicin, different concentrations of doxorubicin were used to treat DLBCL cells. CCK-8 assay was used to detect the proliferation of DLBCL cells. The hsa-miR-28-5p-mimic NC and hsa-miR-28-5p mimic were transfected to doxorubicin-mediated DLBCL cells. Simultaneously, blank control groups were set up. The cells were cultured and transfected for 24 h. Next, each group was administered with different concentrations of doxorubicin and cultured again for 24 h to observe the effects of hsa-miR-28-5p on doxorubicin sensitivity at different times. The proliferation, early apoptosis, and late apoptosis in DLBCL cells were determined using soft agar colony-forming assay, mitochondrial membrane potential assay, and caspase-3 activity assay, respectively. The apoptosis and cell cycle were explored using Annexin V-PE/7-AAD and PI/RNase staining buffer, respectively. We speculated that PD-L1 might be involved in the effect of hsa-miR-28-5p on the sensitivity of adriamycin (doxorubicin) in the DLBCL cells. Hence, we performed immunohistochemistry (IHC) to determine PD-L1 expression within formalin-fixed paraffin-embedded (FFPE) samples from 52 DLBCL cases.

**Results:**

The optimal concentration of doxorubicin targeting DLBCL cells was found to be 3.028 *μ*mol/l. The effect of doxorubicin on DLBCL cells was time- and concentration-dependent. hsa-miR-28-5p mimic + doxorubicin remarkably decreased proliferation of DLBCL. DLBCL cell apoptosis rate was the highest in hsa-miR-28-5p mimic + doxorubicin group. Apart from that, hsa-miR-28-5p mimic plus doxorubicin had the best effect in promoting DLBCL cell apoptosis. After the intervention of hsa-miR-28-5p mimic + doxorubicin on DLBCL cells, the cell cycle was arrested in the S-phase and DNA synthesis was blocked. hsa-miR-28-5p mimic + doxorubicin could regulate the cycle of DLBCL cells. As a result, overexpression of hsa-miR-28-5p combined with doxorubicin is possibly involved in the development of DLBCL by affecting the proliferation, apoptosis, and cycle of DLBCL cells. PD-L1 showed an association with the prognosis of DLBCL patients. Combining with the literature, this suggested hsa-miR-28-5p may influence DLBCL occurrence and therapeutic effect by regulating the PD-L1 level.

**Conclusion:**

The combination of hsa-miR-28-5p mimic and doxorubicin may be considered more effective in inhibiting growth, arresting the cell cycle, and promoting cell apoptosis of DLBCL cells compared to using doxorubicin alone. The effects of doxorubicin on DLBCL cells were found to be time- and concentration-dependent. The overexpression of hsa-miR-28-5p enhanced the effect of doxorubicin on DLBCL cells, which may be attributed to the regulation of PD-L1 levels.

## 1. Introduction

Diffuse large B-cell lymphoma (DLBCL) refers to the most common pathological subtype of non-Hodgkin's lymphoma (NHL) and is the most common type of adult lymphoma, occupying 33.27% [1]. Although regarded as an independent disease by the World Health Organization, DLBCL exhibits great heterogeneity in its clinical features, morphological features, genetic features, immunophenotype, curative effect, long-term prognosis, and so on [1]. Currently, R-CHOP is considered the standard therapy for DLBCL, which includes rituximab (R)-cyclophosphamide (C) + adriamycin (doxorubicin hydrochloride, H) + vincristine (Oncovin, VCR, O) + prednisone (P). The continuous progress of modern radiotherapy, chemotherapy, immunotherapy, and targeted therapy has not only ameliorated the quality of life and the long-term prognosis of DLBCL patients but also has prolonged the progression-free survival and overall survival (OS) rates of such patients. However, due to the individualized difference in the treatment of DLBCL patients and the drug resistance of tumor cells under the constant stimulation of chemotherapy drugs, one-third of patients often relapse and enter the stage of tumor progression shortly after the treatment [2]. In China, the incidence of lymphoma is relatively high, but the OS status is low. Therefore, studying the mechanism of drug resistance in DLBCL can further improve the current treatment method of DLBCL, as well as supply theoretical support to the development of new drugs to extend the OS of lymphoma patients in China. Overall, there is a need to urgently settle the survival of relapsed/refractory (R/R) DLBCL.

Our research group showed that the overexpression of Homo sapiens (hsa)-microRNA (miR)-28-5p inhibited the proliferation, promoted apoptosis, and arrested the cycle of DLBCL cells in the S-phase [3]. However, the effect of hsa-miR-28-5p on the sensitivity of doxorubicin in DLBCL remains unclear.

## 2. Material and Methods

### 2.1. Cells and Culture

Human DLBCL cells: we chose the OCI-LY1 cell line (GCB) in the Institute of Jennio Biosciences (CBP60265, Guangzhou, China) and cultured them within RPMI-1640 medium (C11875500CP/8119428, Gibco, USA) that contained 1% penicillin-streptomycin (PS) (15070-063, 10000U, GIBCO, USA) as well as 10% fetal bovine serum (FBS) (FND500, Excell Bio, USA). All cells were incubated at 37°C in a humidified incubator with 5% CO_2_.

### 2.2. Cell Transfection

The hsa-miR-28-5p mimic (26660, Suzhou, China) and hsa-miR-28-5p mimic negative control (NC) (05215, Suzhou, China) were obtained from Gene Pharma. Lipofectamine 3000® (L3000-008, Invitrogen, USA) was adopted for transfecting the cells as per the manufacturer's instructions. The NC and hsa-miR-28-5p mimics were labeled with red fluorescence (0.1 *μ*m) and then transfected into the cells and incubated for 48 h posttransfection. Red fluorescence intensity was observed with naked eyes with the fluorescence microscope to determine the transfection efficiency, which was determined to be more than 70%.

### 2.3. Cell Counting Kit-8 (CCK-8)

Cell proliferation was practiced with the use of the CCK-8 reagent (N20821, FC101-03, Beijing, China). Seed OCI-LY1 cells into 96-well plates at the density of 5 × 10^3^ cells/well. According to the incubation period, this work added CCK-8 solution (10 *μ*L) to culture OCI-LY1 cells under 37°C for a 1 h period. The microplate reader was then adopted for measuring absorbance (OD) value at 450 nm.

### 2.4. Soft Agar Colony-Forming Assay

OCI-LY1 cells were grown in the indicated conditions. We plated cells in 6-well plates (1.5 mL/well) and cultivated them for a month. Meanwhile, 300 *μ*L of culture medium was added to the plates every three days to avoid drying. Also, the level of cell clone formation was constantly monitored under a microscope. After about a month, the cells were washed with PBS (ZLI-9062, Beijing, China), and the colonies were stained using crystal violet (0.005%, Shanghai, China). The number of cells from each group was compared and analyzed, and the rate of clone formation was calculated. Later, twenty fields of vision were randomly selected and observed under an inverted microscope (100×). The clone formation rate was calculated as the ratio of the number of > 50 clones divided by all clones in the fields of vision scored under a microscope.

### 2.5. Mitochondrial Membrane Potential Assay

Flow cytometry was adopted for detecting mitochondrial membrane potential. Cells were collected and transferred to a centrifuge tube, the mixture was centrifuged at 1000 rpm for 5 min, and then the supernatant was discarded. OCI-LY1 cells were washed twice with cold PBS, and the supernatant was removed. Rhodamine 123 (83702, sigma, USA) with a volume of 500 *μ*L was taken to resuspend these cells with a final concentration of 10 *μ*M. The cells were incubated in an incubator at 37°C for 30 min, washed, and resuspended with PBS. In addition, the fluorescence intensity was measured at the excitation wavelength of 488 nm and the emission wavelength of 529 nm by the flow cytometry, respectively. Finally, FlowJo cytometry analysis software was adopted to analyze early apoptosis in cells of different groups. Meanwhile, it was necessary to ensure the consistency of the pH value in the balanced dye solution during the experiment.

### 2.6. Caspase-3 Activity Assay

The cells were collected in a tube and centrifuged. After centrifugation, the supernatant was discarded and 100 *μ*L of reagent II was supplemented to the pellet based on the number of cells (about 10^6^). The visible spectrophotometer (Nano-100, Hangzhou, China)/Enzyme labeling instrument (xMarkTM, Bio-Rad, USA) was preheated for more than 30 min while the wavelength was adjusted to 405 nm, and the machine was set to zero using distilled water. Next, to prepare the standard curve, the 5 mmol/L PNA reagent was diluted to different concentrations of 200, 100, 50, 25, 12.5, and 0 mmol/L solutions using a standard diluent. Simultaneously, the test sample was also prepared, and the absorbance was measured at 405 nm. The caspase-3 activity was determined with the use of a caspase-3 activity assay kit (BC3830, Beijing, China), following the manufacturer's instructions.

### 2.7. Flow Cytometry Assay

Flow cytometry (LSRFortessa, BD, USA) was applied to analyze the cell cycle. We resuspended cells resuspended in 500 *μ*L of PBS (ZLI-9062, Beijing, China). Meanwhile, 3.5 mL of anhydrous ethanol was used for fixation overnight. The suspension was centrifuged for a 5 min period at 2,000 rpm to separate cells (1 × 10^6^). Next, the cells were rinsed twice with precooled PBS, resuspended in 500 *μ*L of PI/RNase Staining Buffer (550825, BD, USA), and passed sequentially through the 200 *μ*m-mesh nylon sieves to obtain a single-cell suspension. This was followed by 30 min incubation in the dark at 4°C. The samples were then measured within one hour of incubation. The difference in the cell cycle among different groups was compared to understand the distribution of cells at different time points. For apoptosis analysis, collect cells after transfection for 48 h. The Annexin V-PE/7-AAD Kit (9283373, 559763, BD, USA) was employed for cell double-staining and tested after half an hour.

### 2.8. Tissue Samples

The current work was permitted by the Medical Ethics Committees of The Tumor Hospital Affiliated with Xinjiang Medical University and Karamay Central Hospital. We screened 192 patients between January 2010 and December 2021 and finally enrolled 52 patients in the study. All patients were treatment-naive, and each of their samples was fixed in the formalin-fixed paraffin-embedded (FFPE) tissue blocks.  Table 1 presents the characteristics of FFPE tissues obtained from 52 cases of our study.

#### 2.8.1. Pathological Data

*(1) Immunohistochemistry (IHC)*. A fully automatic immunohistochemistry instrument was used for the IHC assay. The antibodies selected for paraffin sections were PD-L1 and SP263 (Roche). DLBCL is highly heterogeneous, i.e., different individuals of the same tumor exhibit different biological characteristics. It is worth determining the cutoff value of PD-L1 (programmed death-ligand 1, also called B7-H1 or CD274) systematically. For example, the melanoma patients treated with Nivolumab showed the ORR (overall response rate; CR: complete remission; PR: partial remission) to be 67% in the 5% positive group, but 19% in the PD-L1 negative group. Even though PD-L1 expression was reported to be significantly correlated with ORR [4], the same cutoff value in patients suffering from non-small-cell lung cancer (NSCLC) suggested that PD-L1 expression was not associated with ORR [5]. Since selecting the cutoff value of PD-L1 is controversial, we used the cutoff score as ≥ 5% for PD-L1 in the present study. The positive standards for CD10 (56C6, Gene company, 1 : 50, Cytomembrane), Bcl-6 (GI191E/A8, ZSBIO, 1 : 80, Nuclei), and MUM-1 (Mum1p, MXBIO, ready to use, Nuclei) were reported to be ≥ 30% [6]. Based on Han's algorithm, DLBCL was further divided into germinal center B-cell (GCB) subtype displaying the MUM1^−^, Bcl-6^+^, CD10^−^ or CD10^+^ phenotype and the non-GCB subtype exhibiting MUM1^+^, CD10^−^, Bcl-6^+^, or Bcl-6^−^ phenotype (including unclassified and ABC subtype in our study).

### 2.9. Follow-Up Visits

During diagnosis, the follow-ups were initiated through phone or hospital visits, which lasted till March 29^th^, 2022. The causes for the termination of the follow-up were also recorded. Overall survival (OS) was deemed as the proportion of the overall number of survivors after the follow-up by the original overall patient numbers. In this study, the original diagnosis was “0,” after which we rated the 1-month survival.

### 2.10. Statistical Analysis

Data processing was carried out using SPSS 23.0 and GraphPad Prism 8.0 software. All data were represented as means ± S.D. Student's *t*-test, one-way ANOVA, and Fisher's exact test were taken with the purpose of fulfilling statistical analysis. *P* < 0.05 was regarded to be of statistical significance.

## 3. Results

### 3.1. After Intervention with Different Concentrations of Doxorubicin, the CCK-8 Test Was Used to Detect the Proliferation of DLBCL Cells to Explore the Most Suitable Concentration of Doxorubicin

At the concentration of 8 *μ*mol/l of doxorubicin, the inhibition rate of OCI-LY1 cell proliferation was found to be 69.313 ± 5.359%, which was significantly higher than the inhibition rates 59.427 ± 4.145%, 39.563 ± 7.350%, 25.340 ± 4.835%, and 17.108 ± 3.957% at 4, 2, 1, and 0.5 *μ*mol/l concentrations, respectively (*P* < 0.05). An increase in the concentration of doxorubicin resulted in a gradual increase in the suppression of the proliferation of OCI-LY1 cells, with significant differences between the groups (*P* < 0.05). The IC50 of doxorubicin used to intervene with OCI-LY1 cells was found to be 3.028 *μ*mol/l for 24 h, which laid a foundation for future experiments. Overall, we found that doxorubicin hindered the proliferation of DLBCL cells, with an increase in the concentration of doxorubicin enhancing the inhibition rate of DLBCL cells (Figures 1 and 2).

### 3.2. The Effect of hsa-miR-28-5p on Doxorubicin Sensitivity in DLBCL Cells

#### 3.2.1. Impact of Different Intervention Times of hsa-miR-28-5p on Doxorubicin Sensitivity in DLBCL Cells

In our study, the survival rate of OCI-LY1 cells in the hsa-miR-28-5p mimic + doxorubicin group (64.272 ± 2.525%) was found to be the lowest after 24 h, with an appreciable difference from that of the control (100 ± 3.163%), doxorubicin (76.533 ± 3.064%), and hsa-miR-28-5p mimic NC + doxorubicin groups (74.448 ± 1.848%) (*P* < 0.05). The cell survival rate of the Control group was different from that of hsa-miR-28-5p mimic NC + doxorubicin and doxorubicin groups, respectively (*P* < 0.05), but there existed no obvious difference between doxorubicin group and hsa-miR-28-5p mimic NC + doxorubicin group (*P* > 0.05). After 48 h of intervention, the survival rate was lowest in the hsa-miR-28-5p mimic + doxorubicin group (39.351 ± 5.9%), with obvious differences between the control (100 ± 7.953%) and hsa-miR-28-5p mimic + doxorubicin groups, doxorubicin (57.478 ± 2.187%) and hsa-miR-28-5p mimic + doxorubicin groups, and also between hsa-miR-28-5p mimic + doxorubicin and hsa-miR-28-5p mimic NC + doxorubicin groups (55.039 ± 1.612%) (*P* < 0.05). The survival rate of cells in the control group was different from that of the doxorubicin group, and hsa-miR-28-5p mimic NC + doxorubicin group (*P* < 0.05), with no obvious difference between doxorubicin and hsa-miR-28-5p mimic NC + doxorubicin groups (*P* > 0.05). After 72 h of intervention, the lowest cell survival was observed in the hsa-miR-28-5p mimic + doxorubicin group (27.216 ± 1.238%), with an unsubtle difference from that of the control (100 ± 3.368%), doxorubicin (46.159 ± 2.187%), and hsa-miR-28-5p mimic NC + doxorubicin groups (43.250 ± 3.060%) (*P* < 0.05). Moreover, clear differences in the cell survival rate were observed between the control and doxorubicin groups, and the control and hsa-miR-28-5p mimic NC ± doxorubicin groups (*P* < 0.05). However, no differences were found between the doxorubicin and hsa-miR-28-5p mimic NC + doxorubicin groups (*P* > 0.05). After 96 h of intervention, the survival rate was observed to be the lowest in the hsa-miR-28-5p mimic + doxorubicin group (14.966 ± 1.678%) compared to that of the control (100 ± 5.933%), doxorubicin (34.592 ± 2.386%), and hsa-miR-28-5p mimic NC + doxorubicin groups (33.764 ± 1.645%) (*P* < 0.05). The cell survival rate of the control group was different from that of hsa-miR-28-5p mimic NC + doxorubicin and doxorubicin groups, respectively (*P* < 0.05), but there was no significant difference between doxorubicin group and hsa-miR-28-5p mimic NC + doxorubicin group (*P* > 0.05) (Figure 2). Overall, we found that the survival rate of DLBCL cells showed a gradual decrease with an increase in the intervention time, with the survival rate being the lowest in the hsa-miR-28-5p mimic + doxorubicin group at an identical intervention time (Figures 3 and 4).

#### 3.2.2. Effect of hsa-miR-28-5p on Doxorubicin Sensitivity in DLBCL Cells with different Intervention Concentrations of Doxorubicin

At the concentration of 8 *μ*mol/l of doxorubicin, the inhibition rate of OCI-LY1 cells was found to be 69.312 ± 5.358% in the control + doxorubicin group, which was different from the inhibition rates of 59.428 ± 4.147%, 39.562 ± 7.348%, 25.34 ± 4.836%, and 17.108 ± 3.959 at 4, 2, 1, and 0.5 *μ*mol/L concentrations, respectively, indicating different inhibition rates of cell proliferation by different concentrations (*P* < 0.05). Similarly, at the doxorubicin concentration of 8 *μ*mol/l, the inhibition rate in the hsa-miR-28-5p mimic NC + doxorubicin group was 74.614 ± 3.947% compared to 62.454 ± 1.911%, 44.83 ± 3.642%, 26.65 ± 3.610%, and 20.492 ± 2.856% at 4, 2, 1, and 0.5 *μ*mol/L concentrations, respectively, exhibiting diverse inhibition rates of cell prolifderation (*P* < 0.05). At the doxorubicin concentration of 8 *μ*mol/l, the inhibition rate in hsa-miR-28-5p mimic + doxorubicin group was 85.554 ± 2.981%, compared to 72.616 ± 5.234%, 64.16 ± 4.378%, 41.216 ± 4.018%, and 29 ± 3.453% at 4, 2, 1, and 0.5 *μ*mol/L concentrations. Different doxorubicin concentrations showed different cell inhibition rates in the hsa-miR-28-5p mimic + doxorubicin group (*P* < 0.05). Thus, we found that with an increase in doxorubicin concentration, the inhibition of DLBCL cell growth became steadily higher (Figures 5 and 6). Also, the hsa-miR-28-5p mimic + doxorubicin group showed the highest inhibition rate on the cell growth of DLBCL at the same intervention concentration of doxorubicin.

### 3.3. Exploration of the Mechanism Underlying the Effect of hsa-miR-28-5p on Doxorubicin Sensitivity in DLBCL Cells

#### 3.3.1. Soft Agar Colony-Forming Assay

The cell clone formation assay determined that the clone cell number of the OCI-LY1 cells in hsa-miR-28-5p mimic + doxorubicin, hsa-miR-28-5p mimic NC + doxorubicin, doxorubicin, and control groups were found to be 17.000 ± 5.568, 31.333 ± 5.508, 33.000 ± 5.000, and 71.667 ± 9.452, respectively. The hsa-miR-28-5p mimic + doxorubicin group displayed the least number of cell clones, exhibiting a statistically significant difference from the other groups (*P* < 0.05). There existed a difference in the number of cell clones between the control group and hsa-miR-28-5p NC + doxorubicin group, and the doxorubicin group, respectively (*P* < 0.05). The difference in the number of cell clones between hsa-miR-28-5p mimic NC + doxorubicin and doxorubicin groups did not appear (*P* > 0.05), which indicated that hsa-miR-28-5p mimic could enhance the inhibiting ability of doxorubicin on the proliferation of OCI-LY1 cells. The final result of this experiment demonstrated that the overexpression of hsa-miR-28-5p could improve the ability of doxorubicin with the purpose of inhibiting the proliferation of DLBCL cells (Figures 7 and 8).

#### 3.3.2. Detection of Mitochondrial Membrane Potential Using Flow Cytometry

The fluorescence intensity of Rhodamine 123 in hsa-miR-28-5p mimic + doxorubicin, hsa-miR-28-5p mimic NC + doxorubicin, doxorubicin, and control groups was found to be 48.226 ± 1.633%, 64.652 ± 3.070, 64.054 ± 2.985%, and 100.000 ± 4.356%, respectively. The fluorescence intensity between the group hsa-miR-28-5p mimic + doxorubicin and the remaining three groups showed a statistical difference (*P* < 0.05).  Also, the intensity between the control and hsa-miR-28-5p mimic NC + doxorubicin group, and the control and doxorubicin groups showed statistical differences (*P* < 0.05). However, no differences were found in the fluorescence intensity between hsa-miR-28-5p mimic NC + doxorubicin and the doxorubicin groups (*P* > 0.05). The lowest fluorescence activity of Rhodamine 123 was observed in the hsa-miR-28-5p mimic + doxorubicin group. Overall, our results showed that upon using doxorubicin alone, the fluorescence intensity of Rhodamine 123 showed a slight decrease, which also indicated a slight decrease in the mitochondrial membrane potential and mitochondrial membrane integrity. However, the combination of hsa-miR-28-5p mimic and doxorubicin showed an obvious decline in the fluorescence intensity of Rhodamine 123. Thus, the visibly decreased mitochondrial membrane potential in the hsa-miR-28-5p mimic + doxorubicin group implied that the combination of both drugs made the tumor cells present with early apoptosis during the treatment of DLBCL (Figure 9).

#### 3.3.3. Caspase-3 Activity Assay

The caspase-3 activities of the cells in the hsa-miR-28-5p mimic + doxorubicin, hsa-miR-28-5p mimic NC + doxorubicin, doxorubicin, and the control groups were found to be 35.463 ± 6.493, 27.374 ± 2.389, 24.327 ± 3.099, and 14.806 ± 2.145 U/mg protein, respectively, exhibiting a gradually decreasing trend. The caspase-3 activity of the hsa-miR-28-5p mimic + doxorubicin group was obviously different, exhibiting the highest apoptotic cell percentage and most potent anti-DLBCL therapeutic effect compared to the remaining three groups. The activity of caspase-3 in the control group, doxorubicin group, hsa-miR-28-5p mimic NC + doxorubicin group, and hsa-miR-28-5p mimic + doxorubicin group increased successively, and the difference of caspase-3 activity between the control group and doxorubicin group, hsa-miR-28-5p mimic NC + doxorubicin and control groups were statistically significant, respectively (*P* < 0.05). It can be seen that doxorubicin enhances DLBCL cell apoptosis. The final results demonstrated that hsa-miR-28-5p mimic could enhance the role of doxorubicin in promoting DLBCL apoptosis (Figure 10).

#### 3.3.4. Impact of the Combination of hsa-miR-28-5p Mimic and Doxorubicin on Apoptosis of DLBCL Cells

The cell apoptosis was examined by flow cytometry. Our results revealed that the percentage of apoptosis in the control, doxorubicin, hsa-miR-28-5p mimic NC + doxorubicin, and hsa-miR-28-5p mimic + doxorubicin groups were found to be 7.827 ± 0.671%, 15.613 ± 0.660%, 15.683 ± 1.292%, and 24.460 ± 1.020%, respectively. Also, the hsa-miR-28-5p mimic doxorubicin group was significantly different from the other groups (*P* < 0.05). The apoptosis rate in control group was different from that of the hsa-miR-28-5p mimic NC + doxorubicin and doxorubicin groups. Early apoptosis rate in the hsa-miR-28-5p mimic + doxorubicin group (15.23%) was found to be higher than that of the control (2.68%), doxorubicin (7.02%), and hsa-miR-28-5p mimic NC + doxorubicin groups (6.51%). Overall, our results suggested that the combination of doxorubicin and hsa-miR-28-5p mimic accelerated the apoptosis of DLBCL cells, improving the therapeutic efficacy of doxorubicin (Figure 11).

#### 3.3.5. Effects of the Combination of hsa-miR-28-5p Mimic and Doxorubicin on the Cell Cycle of DLBCL Cells

The cell cycle was explored using flow cytometry. We found that the cell cycle was arrested at the S-phase in 38.027 ± 0.488%, 21.617 ± 0.635%, 20.440 ± 0.606%, and 15.897 ± 0.225% of cells in the hsa-miR-28-5p mimic + doxorubicin, hsa-miR-28-5p mimic NC + doxorubicin, doxorubicin, and control groups, respectively. The hsa-miR-28-5p mimic + doxorubicin group showed an increased percentage of cells in the S-phase compared to the other three groups (*P* < 0.05). Therefore, the intervention with hsa-miR-28-5p mimic + doxorubicin showed a significant decrease in the cell growth and arrest of the cell cycle in the S-phase, eventually blocking the DNA synthesis in tumor cells. Our results indicated that the hsa-miR-28-5p blocked the replication of OCI-LY1 cells and regulated the transitions among the S, subsequent G2/M, and the previous G0/G1 phases. Simultaneously, the cell proportion in the G0/G1 phase in the hsa-miR-28-5p mimic + doxorubicin group was found to be lower than that of the other three groups (*P* < 0.05). The doxorubicin group had a significantly lower ratio of cells in the G2/M phase than the hsa-miR-28-5p mimic + NC group, but it was more than that in the control group (*P* < 0.05). In addition, the cell percentage of the S-phase in the hsa-miR-28-5p NC + doxorubicin group and doxorubicin group was higher when compared with that in the control group, respectively (*P* < 0.05). The percentage of S-phase cells between hsa-miR-28-5p NC + doxorubicin and doxorubicin groups was different (*P* < 0.05). It could be seen that after doxorubicin intervention, OCI-LY1 cell proliferation decreased, the number of cells in the S-phase increased, and cells were arrested in the S-phase. In addition, the overexpression of hsa-miR-28-5p promoted the ability of doxorubicin to regulate the OCI-LY1 cell cycle, which resulted in the arresting of more OCI-LY1 cells in the S-phase, reducing the proliferative activity of tumor cells (Figure 12).

### 3.4. Relationship between PD-L1 and the Prognosis of Patients in Human DLBCL Tissues

The next goal of our research group was to study whether the effect and mechanism of hsa-miR-28-5p in the occurrence and therapeutic effect of DLBCL was through the regulation of PD-L1 levels. Therefore, to determine the expression levels of PD-L1 in DLBCL tissues, we selected the tissues from the primary central nervous system of DLBCL (PCNS-DLBCL) patients in our experiment, which is shown in Figures 13(a)–13(f). When the cutoff value of PD-L1 was 10% or 20%, PD-L1 was not found connected to the prognosis of DLBCL patients (*P*=0.087 > 0.05 or *P*=0.093 > 0.05), but if the cutoff value was 5%, PD-L1 was found to be associated with a better prognosis of DLBCL patients (*P*=0.043 < 0.05) (Figures 13–14).

## 4. Discussion

Clinically, the primary manifestation of DLBCL is “painless and swollen lymphadenopathy” that usually occurs in the lymph nodes. However, it can also be found in the gastrointestinal tract, liver, skin, lungs, brain, testicles, uterus, ovaries, and other extra-nodal organs. Often the first reason for such patients to go to the doctor is lymphadenopathy in the neck. DLBCL is highly invasive with a short natural course. The CHOP regimen containing Anthracycline drugs is the most classical treatment used for DLBCL. Although few patients with DLBCL can be cured with CHOP, more than 50% of patients develop resistance or may relapse, probably due to the presence of DLBCL cells resistant to the CHOP regimen [7]. This may eventually lead to patients' death due to the chemo-resistant disease [8]. Recently, with the introduction of Rituximab, R-CHOP has been developed and applied as the standard first-line chemotherapy regimen for DLBCL patients, exhibiting significant improvement in the prognosis. However, some patients have still shown the phenomenon of treatment failure, disease progression, or recurrence due to chemotherapy resistance.

The difficulty in treating DLBCL is related to the multidrug resistance of cancer cells. Multidrug Resistance (MDR) denotes the cross-resistance of tumor cells to certain chemotherapeutic drugs, which belong to different classes of drugs with different structures and functions. Tumor cells use MDR as a vital mechanism to escape the attack of chemotherapeutic drugs. Hortobágyi pointed out that the phenomenon of MDR and adverse drug reactions have limited the wide application of Anthracyclines [9]. Currently, the development of MDR is mainly related to the expression of MDR protein, DNA damage and repair, the change of Topoisomerase II activity, the characteristics of stem cells obtained from the tumor, and the changes in metabolism [10]. Therefore, studying the mechanism of drug resistance in tumor cells and improving the sensitivity of tumor cells to chemotherapeutic drugs has now become a hot topic and urgent problem.

According to the literature, the mechanism of doxorubicin involves the following three main aspects [11, 12]: (1) Doxorubicin insertion into the adjacent base pairs of DNA, resulting in DNA chain cleavage and blocking of DNA and mRNA synthesis. (2) Doxorubicin inhibition of Topoisomerase II activity, eventually leading to DNA fragmentation. (3) Doxorubicin induction of the production of free radicals, triggering lipid peroxidation. According to Lim [13], the overexpression of hsa-miR-28-5p was associated with a better prognosis of DLBCL. DLBCL displayed a different miRNA expression profile from that of the benign B-cells, which dysregulated the miRNAs' role in B-cell differentiation and the creation of the lymphocyte. Doxorubicin affected the proliferation, apoptosis, and cell cycle of breast cancer cells [14]. Hence, to improve the efficacy of the current R-CHOP regimen in DLBCL patients, we focused on studying the effect of hsa-miR-28-5p on doxorubicin sensitivity in DLBCL cells.

Our results suggested that the optimal concentration of doxorubicin to treat DLBCL cells was 3.028 *μ*mol/l. At this concentration, the apoptosis of DLBCL cells was enhanced by doxorubicin, and also the DLBCL cells were less resistant to doxorubicin. Doxorubicin is a highly effective chemotherapeutic agent which belongs to the group Anthracyclines. It is also a specific inhibitor of Topoisomerase II, which can inhibit DNA and RNA synthesis. Considered to be one of the most effective chemotherapeutic drugs, doxorubicin is the most widely used Anthracycline drug leading to cytotoxic death of tumor cells. It also exhibits significant chemotherapeutic activity in lymphoma, breast cancer, acute leukemia, and so on [15]. However, the emergence of doxorubicin resistance has limited its application in clinical treatment. Several studies have shown that drug resistance in tumor cells may be associated with miRNAs [16]. miRNAs are speculated to regulate about one-third of human genes. The miRNA regulation in gene expression is an independent feature that distinguishes it from other RNAs, making it a new tumor biomarker and potential therapeutic target [17]. Besides the influence of pharmacological mechanisms, drug resistance in tumors is also related to the abnormal regulation of miRNA on target genes in diseases such as lung cancer, liver cancer, colorectal cancer, and breast cancer [18–21]. Numerous miRNAs are recognized as biomarkers for B-cell lymphoma, with their aberrant levels tightly associated with the disease's occurrence [22, 23]. miRNAs are also found tightly related to the genesis and progression of DLBCL [24]. Studies have reported that miR-34a, miR-99a-5p, miR-125b-5p, miR-155, miR-370-3p, miR-381-3p, and miR-409-3p are abnormally expressed in DLBCL disease [24–27]. miRNAs are a therapeutic target that can add the sensitivity of DLBCL cells to chemotherapy. They are also associated with chemosensitivity in a variety of malignant tumors, including DLBCL [28, 29]. In 2019, Amri identified miR-125a-5p to be a potential therapeutic adjuvant for lung cancer [18]. Overexpression of miR-185 can lead to shorter survival by improving TKI sensitivity in TKI nonresponder stem/progenitor cells [28].

Up-regulation of miR-185 expression is reported to increase the radiosensitivity of colorectal cancer cells [30]. Therefore, it is urgent to study the effect of miRNA inhibitors or miRNA mimics on chemotherapeutic drugs to develop them as auxiliary means of chemotherapy. The above-mentioned studies not only showed the potential clinical value of miRNA as a novel biomarker and therapeutic drug, but they also highlighted the value of miRNA in clinical applications along with their potential in predicting the drug response and applications in treatment.

miR-28, a miRNA, is located within the gene on chromosome 3q28. It is a tumor suppressor and a viral suppressor [31] gene, which is regulated through the binding of STAT5 and p53 to its promoter [32]. In humans, the miR-28 family is divided into subtypes miR-28-3p and miR-28-5p, named after the 3′ and 5′ ends of the pre-miR-28, respectively. These subtypes display biological differences in stability and functionality [33]. Both hsa-miR-28-3p and hsa-miR-28-5p can target several tumor-related genes involved in cell proliferation, migration, invasion, and EMT [34]. The miR-28-5p was reported to be significantly down-regulated in hepatocellular carcinoma [35], colorectal cancer [36], and multiple myeloma [37]. Additionally, miR-28-5p hindered gastric cancer (GC) cell invasion and migration by suppressing NRF2 [38]. It also inhibited the proliferation of nasopharyngeal carcinoma cells in vitro, thus, inducing apoptosis and cell cycle arrest [33]. Moreover, miR-28-5p induced apoptosis of chronic lymphocyte leukemia cells [39] and hindered the proliferation and migration of glioma cells by targeting Rap1b and interfering with genes involved in cell replication and cell cycle checkpoint [40], whose results were consistent with our previous research [3]. Additionally, miR-28-5p inhibited cell proliferation and migration in Renal Cell Carcinoma by directly inhibiting the Rap1b gene [41]. The miR-28-5p was also reported to inhibit cell growth and promote apoptosis of DLBCL cells through Curcumin [42]. Studies have also found that miR-28-5p was upregulated in some tumors, implying their critical role in tumor metastasis and invasion [43]. Besides, the miR-28-5p induced the arrest of ovarian cancer cells in the S-phase by down-regulating N4BP1 along with promoting their proliferation and invasion [34]. A study suggested that miR-28-5p suppressed the cell growth, invasion, and migration of NSCLC by targeting HIF-1*α* and inducing apoptosis in lung cancer cells [44].

The miR-197 mimic can enhance the chemosensitivity of lung cancer cells by increasing the PD-L1 expression [29]. The miRNAs can promote the efficacy of NSCLC by modulating PD-L1 levels and other molecules involved in cell proliferation [45, 46]. In the current work, we found that positive expression of PD-L1 in DLBCL tissues was related to a good prognosis of DLBCL patients at the cutoff value of 5%, which was similar to a related study [47]. However, it was inconsistent with some other studies [48]. Our research group aims to explore the expression levels of PD-L1 in DLBCL cells and also the mechanism underlying the effect of hsa-miR-28-5p on the development and therapeutic effect of DLBCL through the regulation of PD-L1 expression.

## 5. Conclusion

In summary, the combination of hsa-miR-28-5p and doxorubicin is more effective than doxorubicin alone in inhibiting cell proliferation, promoting apoptosis, and blocking the cell cycle of DLBCL cells. Also, the effects of doxorubicin on DLBCL cells were found to be time-and concentration-dependent. Overexpression of hsa-miR-28-5p enhances the therapeutic effect of doxorubicin on DLBCL cells, which may be attributed to its role in modulating the PD-L1 levels. Our findings may provide a new treatment method to reduce the multidrug resistance in DLBCL cells, laying a foundation for the next step of future research.

## Figures and Tables

**Figure 1:** Images of doxorubicin interfering with the proliferation of OCI-LY1 cells (100x).

**Figure 2:** Effect of doxorubicin on the proliferation of OCI-LY1 cells. ^*∗*^*P* < 0.05 vs. doxorubicin (0.5 *μ*M) group; ^#^*P* < 0.05 vs. doxorubicin (1 *μ*M) group; ^&^*P* < 0.05 vs. doxorubicin (2 *μ*M) group; °*P* < 0.05 vs. doxorubicin (4 *μ*M) group.

**Figure 3:** The survival rate of OCI-LY1 cells in different groups at varying intervention times. ^*∗*^*P* < 0.05,^#^*P* < 0.05,^&^*P* < 0.05 vs. control, doxorubicin, and hsa-miR-28-5p mimic NC + doxorubicin groups, separately.

**Figure 4:** The images of OCI-LY1 cells in different groups at different intervention times (100x).

**Figure 5:** Images of OCI-LY1 cells in different groups treated with different concentrations of doxorubicin (100x).

**Figure 6:** The proliferation of OCI-LY1 cells in different groups treated with different concentrations of doxorubicin. ^*∗*^*P* < 0.05 vs. doxorubicin (0.5 *μ*M) group; ^#^*P* < 0.05 vs. doxorubicin (1 *μ*M) group; ^&^*P* < 0.05 vs. doxorubicin (2 *μ*M) group; °*P* < 0.05 vs. doxorubicin (4 *μ*M) group.

**Figure 7:** Images of cell clone formation in the OCI-LY1 cells (100x). (a) Control. (b) Doxorubicin. (c) Mimic NC + doxorubicin. (d) Mimic + doxorubicin.

**Figure 8:** Effects of different interventions on the cell clone numbers of OCI-LY1 cells. ^*∗*^*P* < 0.05 vs. control group; ^#^*P* < 0.05 vs. doxorubicin group; ^&^*P* < 0.05 vs. hsa-miR-28-5p mimic NC + doxorubicin group.

**Figure 9:** Flow and column diagrams of fluorescence detection of Rhodamine 123. ^*∗*^*P* < 0.05 vs. control group; ^#^*P* < 0.05 vs. doxorubicin group; ^&^*P* < 0.05 vs. hsa-miR-28-5p mimic NC + doxorubicin group.

**Figure 10:** Effects of different interventions on the activity of caspase-3. ^*∗*^*P* < 0.05 vs. control group; ^#^*P* < 0.05 vs. doxorubicin group; ^&^*P* < 0.05 vs. hsa-miR-28-5p mimic NC + doxorubicin group.

**Figure 11:** Effects of the combination of hsa-miR-28-5p and doxorubicin on the apoptosis of OCI-LY1 cells. (a) Flow cytometry detection of apoptosis; (b) statistical analysis graph; (c) the expression of apoptosis-related proteins detected by WB. ^*∗*^*P* < 0.05 vs. control group; ^#^*P* < 0.05 vs. doxorubicin group; ^&^*P* < 0.05 vs. hsa-miR-28-5p mimic NC + doxorubicin group.

**Figure 12:** Effects of the combination of hsa-miR-28-5p and doxorubicin on the cell cycle of OCI-LY1 cells.

**Figure 13:** Immunohistochemical results of DLBCL tissues (diffuse large B-cell lymphoma) (EnVision method, original magnification 200x). (a) Negative control; (b) PD-L1-negative oncocytes; (c) positive control: PD-L1 expression in placental tissue; (d) PD-L1 weak positive expression in oncocytes; (e) PD-L1 moderate positive expression in oncocytes; (f) PD-L1 strong positive expression in oncocytes.

**Figure 14:** Univariate analysis of DLBCL patients in various groups. (a) 5% cutoff value of PD-L1; (b) 10% cutoff value of PD-L1; (c) 20% cutoff value of PD-L1.

**Table 1:** Characteristics of 52 DLBCL patients used for the preparation of FFPE tissue samples.

Item	GCB group	Non-GCB group	*P* value
*n*	17	35	—
Age (years), *n* (%)			
≤60	5 [5/17, 29]	19 [19/35, 54]	0.091
>60	12 [12/17, 71]	16 [16/35, 46]	
Gender, *n* (%)			
Male	7 [7/17, 41]	15 [15/35, 43]	0.908
Female	10 [10/17, 59]	20 [20/35, 57]	
Laboratory parameter, mean ± SD (10^9^/l)			
Neutrophil granulocyte	5.62 ± 3.13	4.89 ± 2.58	0.079
Monocyte	0.49 ± 0.19	0.59 ± 0.05	0.445
Thrombocyte	219.94 ± 51.76	225.4 ± 71.74	0.735
LDH, *n* (%)			
Increased	4 [4/17, 24]	8 [8/35, 23]	0.957
Decreased	13 [13/17, 76]	27 [27/35, 77]	
Ki67, *n* (%)			
≥ 70%	15 (15/17, 88)	29 (29/35, 82)	0.707
< 70%	2 (2/17, 12)	6 (6/35, 17)	
Treatment options, *n* (%)			
Operation or chemotherapy	14 [14/17, 82]	26 [26/35, 74]	0.517
Comprehensive treatment	3 [3/17, 18]	9 [9/35, 26]	
Overall survival (%)	7 [7/17, 41]	13 [13/35, 37]	0.779

## Data Availability

All data generated or analyzed during this study are included in this published article.
